This article has been retracted.

# Changing Positive Academic Emotions of Art Students Utilizing Computer Information Technology Based on the Perspective of Teaching

**DOI:** 10.1155/2022/7184274

**Published:** 2022-06-14

**Authors:** Yihong Sun

**Affiliations:** School of Public Education, Shandong College of Arts, Jinan 250014, Shandong Province, China

## Abstract

This study is aimed at exploring the influencing factors on the altering academic mood of art students. With the assistance of computer information technology, the survey utilizing a questionnaire is conducted to explore the influence of different coping styles on the academic moods of art students when the influence of demographic variables is under consideration. It is concluded that the condition of being the only child of art students has a positive and high arousal emotional score of 80.93, which is significantly higher than that of not being an only-child art student of 78.61. Art students are more inclined to take a positive coping style. The scores of negative and high arousal academic emotions are found to be 79.3, 80, and 96.83, respectively, when the grade changes from 1 through 3. The general trend is that the scores of negative and high arousal academic emotions increase when grades go up. Art students experience more negative academic emotions than positive academic emotions when the general characteristics of art students' academic emotions are under consideration. Because females are more sensitive and delicate, they experience more negative academic emotions. Besides, while a positive coping style can positively predict art students' positive academic mood, a negative coping style can positively estimate the negative academic mood. It is concluded that the outcomes could provide a reference for the prediction of academic mood changes in art students.

## 1. Introduction

As a special group of students, art students should not only study professional courses but also cultivate artistic literacy. Thus, coping with both will cause art students to have a lot of academic burdens. [1] found that when the academic burden is compared between primary and high school students in China, it increases as the academic level does too. Besides, when the academic burden is compared between basic and higher education students in a solid setting, students at the universities have to deal with more than do both primary and high school students. Moreover, this hectic state will add negative emotions such as a feeling of being lost, frustration, learning anxiety, and depression to their learning efforts, resulting in unstable academic performance, low enthusiasm for learning new things, blurry learning goals, and even academic burnout eventually. How to make art students comprehend and evaluate themselves correctly, enhance self-confidence, improve concentration on studies, and maintain a good academic mood is worthy of social thinking [2].

The sign that academic emotion has reached a new level in research is as follows: the magazine titled *Educational Psychologist* in 2002, Volume 37 (No. 2) selected 8 articles related to the research of academic emotion. Those articles examine academic emotions from different perspectives such as academic achievement and learning motivation [3]. At present, the research results on academic emotion have two aspects: (1) academic emotion and learning motivation: students' willingness, effort, and motivation are related to academic emotions. On the other hand, negative academic emotions such as anger and disappointment could affect the motivations of students to learn. However, there could be some exceptions for example being ashamed. In contrast, these kinds of negative emotions could also enhance the learning initiatives of students so that they could achieve great progress in their learning efforts [4]. Interest, motivation, strategies of learning, and internal versus external control of regulation under the title of self-regulated learning of students that are very closely related to emotions predict achievements in an academic setting. So, considering emotions is crucial. Instead categorizing negative one as a deterrent and positive one as promotional is not a good approach since sometimes the opposite effect could occur [5].

(2) Academic emotion and attribution: human beings experience pride when they attribute success to internal factors but feel shame when they fail. Different attribution methods would make human beings have different emotional experiences. Relating attributions to the associated specific emotions could not be conducted easily since both positive and negative ones could lead to, are extensively thought prevalent and dominant patterns but not unique ones. When compared, negative emotions are more differentiated than positive emotions [6]

At present, researchers in China pay more attention to the status quo of academic emotions, but most of them are limited to searching for differences concerning demographic variables, and the research results are not the same [7]. Moreover, the main points of research on the current situation of academic emotions for ordinary college students are as follows: there exist differences concerning both gender and source of students in the academic emotions of college students. There also exist significant differences in gender and grade in academic mood, but no significant difference is found in origin. Besides, the academic mood of college students has important differences in grades, for example, freshmen have the highest academic mood score. Accordingly, college students have a higher academic emotional experience when they deal with the pleasant category, for example, females studying liberal arts are more pleasant than males studying liberal arts. Even though the outcomes of gender on emotions have mixed implications, gender is found to be a significant factor [8–11]. So, gender and major are two significant attributes to make significant differences in academic emotions [12].

Currently, there has been limited research on styles of coping and academic emotions together. Both positive and negative styles of coping could predict the occurrence of anxiety and depression. While negative styles of coping could lead to the generation and aggravation of anxiety and depression, positive styles of coping could reduce the occurrence and severity of anxiety and depression. The research on styles of coping and emotions of stressors does not involve the study of academic emotions comprehensively but only focuses on the study of negative emotions. Some of the coping styles with stress sources to emotions regarding higher education students are as follows: In this article, computer information technology (CIT) is employed to explore the influence of different styles of coping on academic mood and to provide a reference for the prediction of academic mood alterations of art students.

## 2. An Overview of the Relevant Theories and the Flow of Research Ideas

### 2.1. Computer Information Technology

The world's first electronic computer was introduced in February of 1946. In the next coming half-century, computers and the Internet gradually moved from experimental phases to implementation stages. The application of computer technology has expanded from the management of initial military scientific research to any field around the globe [13]. Moreover, the Internet merges the entire online world into one giant supercomputer. Then, computers start to realize the comprehensive sharing of computing, communication, software, storage, and information resources. Computer information technology (CIT) has penetrated every corner of life. If there is a computer or a mobile phone, no matter where the person is, connection to any corner of the world is easier than before. In the 21st century, every single site in the world has stepped into the information society. Therefore, the first requirement for a person to be successful is to master the CIT [14, 15].

Education, as a part of society, has also changed with the rise of computing technology. At the end of the 20th century, information technology combined with a computer as the main feature was widely used in both education and the teaching process. Education itself has undergone fundamental changes regarding the purpose, form, content, and method of the organization. The essence of this shift is to require the integration of the CIT with the content of the education.

The integration of computer technology with the content of education is the process called education informatization. In this process, the CIT is utilized extensively and deeply to promote educational reform and development. In conventional teaching activities, teachers are the main skeleton of teaching activities. Thus, the knowledge provided by teachers to students. However, the new teaching concept is that teachers could be the guides and helpers for the learning activities of students and knowledge could be self-constructed by students according to the cognitive structure in their minds. Consequently, this is a brand new teaching concept suitable for guiding, teaching, and learning when an information technology environment is under consideration. With the popularization and application of the CIT, the powerful functions based on the computer network have brought unprecedented convenience and speed to the education provided in schools and the management of teaching [16, 17]. The specific advantages of the CIT are summarized in Figure 1 as follows.

As Figure 1 implies, computer technology combined with customized software and related educational material could help improve the processes of teaching and learning by devising new communication and sharing means such as online courses, more e-based materials, and more effective question-answer sessions. Thus, these types of activities help students more engage in learning activities that result in better positive emotions or less negative emotions.

### 2.2. Academic Mood

In the theory of academic emotions, emotions have always played an important role in the research process of educational psychology. Scholars have been studying the subject since the 1930s, and it was not until 2002 that the concept of academic emotion was first explicitly proposed. Therefore, academic emotions were defined as emotions that are directly related to academic learning, classroom teaching, and academic achievement [18]. With the further enhancement of the concept of academic emotion, scholars believe that academic emotion refers to various emotional experiences related to the academic effort of a student when teaching or learning, including happiness, boredom, disappointment, anxiety, and anger is in progress. It not only refers to the various emotions that students experience after learning of academic success or failure but also includes the emotional experiences of students in classroom learning, in the process of daily homework, and during exams [19].

In the dimension of academic emotion, scholars generally employ pleasure to divide academic emotion such as positive emotion and negative emotion, or the division of positive emotion, neutral emotion, and negative emotion [20]. However, the previous method of classifying academic emotions concerning only pleasantness ignored the dimension of arousal. Therefore, late scholars added arousal to the classification of academic emotions. Besides, academic emotions are divided into four categories: positive high arousal, positive low arousal, negative high arousal, and negative low arousal. While the first category is emotions caused by positive events, the second category is the emotion that occurs when a negative process stops. Moreover, the third category is negative emotions that lack subjective control. Finally, the fourth type of emotion is characterized by a relatively high level of control [21, 22]. The specific performance of the four dimensions of academic emotion is depicted in Figure 2.

The dimension numbers changing between 6 and 10 are suggested to represent academic emotions in the literature. However, it is possible to represent them with a lower number of dimensions. [23] suggested a circumplex model. Nevertheless, the dimensions of organizing emotions remained controversial. When self-reported data is under consideration, emotions can be represented in a two-dimensional setting. While the horizontal line denotes positive vs. negative, the vertical line denotes high vs. low [23].

In the measurement of academic emotions, currently, there have been limited tools to measure academic emotions in China. Three types of scales are frequently employed. The first is called the Academic Mood Questionnaire compiled concerning the Test Anxiety Scale. It consists of three subscales, questionnaires related to study, classroom, and examination. Each subscale includes pride, joy, hope, ease, anxiety, anger, disappointment, shame, and boredom. The second is called the Adolescent Academic Mood Questionnaire consisting of a total of 72 items. It includes 13 different academic emotions, which are divided into four dimensions: positive high arousal, positive low arousal, negative high arousal, and negative low arousal. The third is called the *General Academic Sentiment Questionnaire for College Students*. It contains the academic activities of college students in various fields, and the 88 projects compiled are general. The ten subtests reflect ten emotions, which are further divided into positive high arousals such as interest, sneakiness, hope, negative high arousal such as shame, anxiety, anger, positive low arousal such as pride and relaxation, and negative low arousal such as disappointment and anger [24, 25].

In the influencing factors of academic mood, there exist two categories of factors affecting academic mood in addition to demographic variables: individual internal factors and external environmental factors [26, 27]. The specific performance of these two factors is presented in Figure 3.

In the CIT-based research on academic emotions, empathy could reduce negative emotions such as anger and frustration that learners encounter when utilizing computers to learn. For example, humor removes negative emotions such as anxiety, stress, or tension that students may experience while studying. Therefore, computer technology can be utilized to design a learning system containing an emotional interaction mechanism, which could help students improve their academic mood [28].

### 2.3. Research Ideas and Processes

The process of this questionnaire survey is presented in Figure 4.

(1) Research objects: in this survey, the questionnaire randomly selected 350 art students from a city's art colleges as the research objects, and distributed the questionnaires
(2) Selection of research tools: the *General Academic Emotions Questionnaire of College Students* is employed as a research tool [29]. It includes a total of 88 items and 10 sub-tests. For example, some of the questions are expressed as follows: “I am always nervous when I am approaching the exam,” “I want to sleep as soon as I study,” and “Studying makes me happy.” The scoring method adopts a multilevel scoring method. The specific grades are depicted in Figure 5
(3) Reliability test: reliability refers to the analysis of the same event under the condition that the research method does not change [30]. If the results do not change, it means that the survey results have high reliability, so it can also be called reliability analysis [31]. At present, the commonly used reliability measure is called Cronbach's. Its formula is presented in
  (1) $$\begin{array}{c} \alpha =\frac{K}{K-1}\left(1-\frac{\sum_{i=1}^{K}\sigma_{Y^{i}}^{2}}{\sigma_{X}^{2}}\right), \end{array}$$
  where *K* refers to the total number of questions in the questionnaire, *σ*_*X*_^2^ refers to the variance of the total sample, *σ*_*Y*^*i*^_^2^ refers to the variance of the measurement sample. Statistical Product and Service Solutions (SPSS) software version 25.0 is conducted to analyze the data obtained by running the survey of the questionnaire, and the value of *α* changes between 0 and 1. If 0.9 < *α* < 1, it indicates that the survey results lead to high reliability. If 0.8 < *α* < 0.9, it is an acceptable outcome and the questionnaire can be used for the research problem. If 0.7 < *α* < 0.8, indicates that the reliability of the survey results is low, and it needs to be modified accordingly.
(4) Test and statistical methods: this test is conducted by employing statistical answering. The answering time is about 1 hour, and the questionnaires are collected on the spot. SPSS 25.0 software is conducted to record and organize the whole data, and run to extract descriptive statistics the results of independent sample *t*-test, variance analysis, correlation analysis, regression analysis, and other analyses

## 3. Experimental Results

### 3.1. Statistical Results of the Questionnaire

A total of 350 questionnaires are distributed, and 334 questionnaires are recovered, with a recovery rate of 95.4%. The returned questionnaires are checked, and those that contain missing values are not included in the analysis. Finally, the effective sample rate reached 92.8% (310 fully answered questionnaires) The specific demographic results are presented in Figure 6.

The results of the demographic variables are presented with three perspectives called gender, grade, and whether they are the only child, respectively, in Figures 6(a)–6(c)). While males account for 59.4%, females represent 40.6%, which represents relatively a close ratio between males and females presented in Figure 6(a). While the cases of the single child accounted for 31.3%, the cases of not being the only child accounted for 68.7% presented in Figure 6(b). Once the grade increases, the level of coping with emotions grows lower, presented in Figure 6(c). There exists a sharp decrease between grade 1 and grade 3 when coping with emotions is under investigation, which shows a good agreement with the literature.

### 3.2. The Analysis of the Survey Results

#### 3.2.1. Questionnaire Reliability

The coefficient values of the questionnaire and each subtest are between 0.641 and 0.887, and the consistency reliability is 0.851, which is greater than 0.6 showing a moderate correlation. The College Students' Academic Emotion Questionnaire is an assessment tool that can reflect the characteristics of college students' academic emotions and meet the requirements of psychometrics.

#### 3.2.2. Gender Differences in Art Students' Coping Styles and Academic Emotions

An independent sample *t*-test is conducted on the academic emotions and coping styles of art students concerning genders. The results are depicted in Figure 7.

While the score of males studying art is found to be 63.6, the score of females studying art is found to be 68.4. Males studying art are significantly lower than females, which are presented in Figure 7 concerning negative and low arousal emotions. While the score of males studying art is found to be 57.56, the score of females studying art is found to be 52.31. Males studying art are significantly higher than females studying art. In terms of coping styles, art students generally tend to adopt positive coping styles. Moreover, males studying art are significantly higher than females.

#### 3.2.3. Differences in the Academic Mood and Coping Style of Art Students Whether They Are the Only Children

An independent sample *t*-test is carried out on the academic mood and coping style of art students who were the only children or not. The specific results are depicted in Figure 8.

There exist a significant difference in academic mood between the only child and the not being an only child of art students in Figure 8. While the score of negative and low arousal emotion of the only-child art students is found to be 62.7, which is significantly lower than the score of 66.23 for the not being an only-child art student. The only-child art students' positive and high arousal emotional academic score is found to be 80.93, which is significantly higher than the not being an-only-child art students' score of 78.61. So, there exist no statistically significant differences when the styles of coping are under consideration.

#### 3.2.4. Differences in Grades of Art Students' Academic Emotions and Coping Styles

One-way analysis of variance (ANOVA) is conducted on the academic mood and coping styles of art students concerning different grades. The specific results are presented in Figure 9.

There exist significant differences in the academic emotional dimensions of negative high arousal, negative low arousal, and positive low arousal among art students. The scores of negative and high arousal academic emotions are found to be 79.3, 80, and 96.83, respectively, when grades change from 1 through 3. The overall change trend is expressed as follows: the scores of negative and high arousal academic emotions increase with the grade, which is like the changing trend of negative and low arousal academic emotions. The scores for positive high arousal and positive low arousal academic mood decreased with grade. In terms of coping style, art students of different grades have no significant difference in adopting the positive coping style and negative coping style.

#### 3.2.5. Correlation and Regression Analysis concerning the Styles of Coping and Academic Emotions of Art Students

To examine the relationship between the styles of coping for art students and their academic emotions, the data are employed to conduct correlation analysis and regression analysis, which are depicted in Figure 10.

The correlation analysis between the positive coping styles of art students and the academic emotions of negative high arousal and negative low arousal is found to be 0.176 and 0.208, respectively, showing a significant positive correlation represented in Figure 10(a). Besides, the correlation analysis between the positive coping methods of art students and the academic emotions of positive low arousal and positive high arousal is found to be -0.336, -0.183, showing a significant negative correlation. So, the art students' negative coping styles are negatively correlated with positive and low arousal academic emotions and are significantly positively correlated with negative high arousal and negative low arousal academic emotions, respectively. The predictive effect of positive coping style type and negative coping style type is found to be not significant, which is presented in Figure 10(b) when the regression analysis chooses the positive low arousal as the dependent variable. On the other hand, the regression analysis with negative and high arousal as the dependent variable resulted in the type of positive coping style having a significant predictive effect on it.

## 4. Conclusion

When art students face pressure, applying different coping styles directly has an impact on the academic mood of vocational students. If they would choose a positive coping style, their psychology will develop positively and it is healthy. With the growing number of art students, the research on subjects such as stress, academic emotions, and coping styles of art students carry great value. This research employs a survey based on a questionnaire to explore the impacts of different coping styles on academic mood when demographic variables are under consideration. The outcomes of the experiment show that the only child art students have positive and high arousal emotional scores of 80.93, which is significantly higher than that of not being an only-child art student with 78.61. Thus, art students are more inclined to take a positive coping style. The scores of negative and high arousal academic emotions are found to be 79.3, 80, and 96.83, respectively, when the grade changes from 1 through 3. So, the overall change trend is expressed as follows: the scores of negative and high arousal academic emotions increase with the grade, which is like the changing trend of negative and low arousal academic emotions. Art students experience more negative academic emotions than positive academic emotions when the general characteristics of art students' academic emotions are a concern. Females are found to be more sensitive and delicate and experience more negative academic emotions. Besides, while positive coping styles can positively predict the positive academic mood of art students, negative coping styles can positively predict negative academic emotions. Moreover, coping styles play a moderating role in the impact of positive and low arousal academic emotions. Accordingly, positive coping styles play a moderating role in the effects of negative and high arousal academic emotions. Therefore, cultivating a positive coping style is one of the efficient ways to prevent and overcome the negative academic emotions of students. The limitations of this research include those issues: (1) The picked sample is based on a certain city's art college, and the coverage is not large enough to derive generalized outcomes. More comprehensive samples are planned to be chosen in future research to conduct large-scale research to generate more covering outcomes on this topic.

## Figures and Tables

**Figure 1:** The advantages of the computer technology in the education.

**Figure 2:** The specific manifestations of the academic emotions in four dimensions.

**Figure 3:** The specific performance of both internal and external factors.

**Figure 4:** The framework of the research ideas.

**Figure 5:** The rating scale of a questionnaire.

**Figure 6:** The composition of the test subjects. ((a) gender composition, (b) only child, and (c) grade composition).

**Figure 7:** Differences in academic emotions and coping styles among art students concerning genders ((a) score statistics for each dimension and (b) *t*-test results for each dimension).

**Figure 8:** Differences in academic emotions and coping styles of art students who are the only children or not ((a) score statistics for each dimension and (b) *t*-test results for each dimension).

**Figure 9:** Differences in academic emotions and coping styles of art students in different grades ((a) score statistics for each dimension and (b) one-way analysis of variance for each dimension).

**Figure 10:** The analysis of the types of coping styles and academic emotions of art students ((a) correlation analysis between coping style types and academic emotions and (b) regression analysis between coping style types and academic emotions).

## Data Availability

Data will be provided upon request to the authors.
